RETRACTED

# Characteristics, Experience, and Enlightenment of Leisure and Sports Policy and Public Health Development in Developed Countries

**DOI:** 10.1155/2022/9162584

**Published:** 2022-08-25

**Authors:** Rui Xue, Haogen Li

**Affiliations:** Department of Physical Education, Kunsan National University, Kunsan 541150, Republic of Korea

## Abstract

Public health highlights “public utilities,” emphasizes the attributes of public goods and services, and aims to clarify the responsibility of government leadership; highlighting “maintaining health equity” aims to make it clear that public health not only guarantees health but also focuses on fairness; the purpose extends to “maintaining social stability and development,” emphasizing that the function of public health is not only to protect health; emphasizing that public health is “one science” and aims to call for respect for the laws of science and the cross-integration of medicine with other natural and social sciences; and emphasizing that public health “focuses on practice” makes it clear that strengthening the implementation of various policies and measures is the key to achieving purpose and values. The development of the entertainment and sports industry is directly related to the development, stability, and people's welfare of the country. Under the common influence of various factors, such as the increasing level of social economy and technology, the growth of people's leisure time, and the change in social consumption concept, the development of China's entertainment and sports industry has shown a certain scale effect, social correlation effect, and employment effect. However, due to the continuous advancement of the development process of China's entertainment and sports industry, some problems have emerged, such as uneven development speed, small industrial scale, low industrial technology level, lack of service commodity types, unreasonable market resource allocation, and serious shortage of professionals in relevant fields. Thus, it limits the development process of China's entertainment and sports industry and is not conducive to the ecological development of China's entertainment and sports industry. On this basis, the state has formulated the guiding opinions on improving China's leisure sports policies and regulations: adjusting the method, intensity, and direction of the state's direct financial investment; strengthening the support for social funds and sports clubs; reducing the price and reducing the cost of entertainment; and establishing a reasonable industrial integrity system and standards; a government supervision and performance evaluation system has been initially formed. It aims to highlight that all aspects of society should also serve health while enjoying health; comprehensive policies are the guarantee for promoting the benign operation of the system.

RETRACTED

## 1. Introduction

Sports has played a significant role in the development process of our country, and it can also enable the public to achieve the goal of happy body, self-improvement, and self-cultivation [1] At present, China's leisure sports industry has ushered in a favorable development condition: from the economic point of view, as proposed in the communique of the 19th National Congress of the Communist Party of China, China's economic and social contradictions have begun to shift from “material and cultural needs” to “normal life needs,” and people's income levels have increased significantly [2]. The consumption concept has changed from advocating diet and clothing to advocating health and happiness and other higher levels [3]. It focuses on the continuous increase in the proportion of entertainment, sports, and cultural consumption in per capita disposable income in China, creating a favorable financial environment for the vigorous development of the entertainment, sports, and cultural industry; the improvement of efficiency has released the rural surplus labor force, and the people have more free time to spend. It also provides financial guarantee and support for the healthy development of leisure sports industry; in this context, the manufacturing industry, service industry, and other fields have also received the attention of government departments, which has greatly promoted the vigorous development of leisure sports industry [4]. The characteristics of leisure sports in various places in China are shown in Figure 1 [5]. In 2016, the government office of the State Council issued several opinions on guiding the development of fitness and leisure products and, in 2017 and 2018, the notice on promoting the construction of sports and leisure characteristic towns [6]. This provides an important institutional guarantee for the development of modern leisure sports industry [7].

With the development of the times, its definition should be further elaborated and explained, and “public health” should be replaced and covered with “public health” to better express its profound connotation changes, as detailed in this issue of “From Public Health to Public Health: Historical Inheritance and Development.” Public health needs to rely on the public health system to carry and implement, and the establishment and improvement of the public health system further expand the connotation of public health, and the two complement each other. At present, the definition and connotation of the public health system are different, and the perspectives and starting points are also different. Leisure sports emphasize that the main purpose of all participants is entertainment, leisure, and entertainment and health promotion [8]. Leisure sports environment refers to the general synthesis of various conditions of the main body of leisure sports activities. It can include two types: chemical material environmental protection conditions (hard environmental protection conditions) and nonmaterial environmental conditions (soft environmental protection conditions) [9]. The latter mainly involves economic, technical conditions, economic and social policy environment, political and ideological conditions, population environment, etc. [10]. The conditions of leisure sports include various laws, regulations, and measures formulated in leisure sports and the complex environment formed by their implementation. After entering the 21st century, the world health crisis has become increasingly prominent: the health quality of children and adolescents in the world is generally low, and the obesity rate continues to rise; the impact of network and mobile on health is increasing; the risks and problems of aging society are increasing day by day [11]. To cope with the economic crisis, the state has issued many preferential policies, trying to improve the proportion of sports population and the per capita participation rate of sports health [12]. Although China faces the above risks, unlike developed countries, China's leisure sports industry still maintains a strong growth period with great potential [13]. There are many reasons to promote the vigorous development of leisure sports, such as the improvement of people's income, the development of sports concepts and habits, the improvement of people's pension and medical level, and the relief of educational pressure. One of the reasons is the change in leisure sports policy environment [14]. The healthy and rapid development of leisure sports in China depends more on top-level design. The starting point and significance of this study are to summarize the successful experience of developed countries, improve the policy environment of leisure sports, and promote the healthy and rapid development of leisure sports in China.

RETRACTED

## 2. Theoretical Research

### 2.1. Elaboration of the Concept of Public Health

Public health undertakings, also known as public health services, are undertakings aimed at ensuring the health level of citizens and ensuring social health and equity. Government leadership, community cooperation, active participation, and joint efforts of all community members prevent and control chronic diseases and disabilities using health-related theories and methods, so as to reduce and eliminate health risks and improve and promote the physical and mental health of the whole people, which is the basis for creating a healthy country (region). Mental health education and community adaptation will further improve the physical health level and quality of life of the whole people, to improve the health level and quality of life of the whole people and maintain social stability and development. The proposal of “public health” reflects the historical inheritance and development of five aspects of public health, namely, from the early standardization of personal hygiene behaviors to the improvement of environmental health and the promotion of group health; expand from simple prevention and control of infectious diseases to comprehensive prevention and treatment of various diseases; from reducing disease hazards to reducing health risks throughout the life cycle; from focusing on physical health to valuing mental health to improving social resilience; and shift from passive disease control measures to proactive health risk interventions.

The essential attribute of public health is the public service that brings health to the public and its associated well-being. Related services have public goods attributes, such as noncompetitive and nonexclusive. Nonexclusivity means that no one will be excluded from the consumption of public goods; noncompetitive means that increased consumption does not reduce the satisfaction of others or increase the input of resources. The problems that arise in the development of public health are often closely related to fairness or even the problem of fairness itself. Therefore, it is necessary to emphasize the purpose of maintaining health equity on the basis of ensuring the level of health. The indivisibility of the utility of public health itself also necessarily requires attention to equity, which should be shared by all. Health equity is also an important component of social equity, and all people have the right to “realize their full health potential” and no one can lose this opportunity due to income, social status, and other social factors. In general, health equity encompasses both outcome equity and equity of opportunity, and health inequality is unacceptable at the political, social, and economic levels.

### 2.2. Explanation of the Concept of Leisure Sports

The academic definition of the concept of leisure sports mainly includes the following viewpoints:

1. Emphasizing that leisure sports is a kind of physical activity: Liu Yimin put forward the concept of “leisure sports” (also known as leisure sports) based on the time perspective of people's participation in sports activities [15]. To meet the purpose of recreation, entertainment, fitness, catharsis, and stimulation of various forms of physical activity, its characteristics include the free choice of individuals, the comprehensiveness of activity values, and the diversity of activity forms and contents [16]. He emphasized that leisure sports cover recreational sports, fitness sports, and medical rehabilitation sports [17]. Tian Hui and Zhou Hong define leisure sports as follows: “all kinds of sports activities that people do in their spare time to achieve physical health and psychological pleasure” and believe that leisure sports has a variety of sports forms, a wide range of service objects and functional universality, and other characteristics; Table 1 describes the characteristics of different leisure sports types. Qiu Yajun believes that leisure sports are carried out in leisure time, to achieve the purpose of entertainment, fitness, recreation, and stimulation and to pursue a positive experience of physical activity [18]. The experience of leisure sports includes physical, psychological, sociocultural, aesthetic, and recreational [19].
2. Emphasizing that the purpose of leisure sports is emotional experience: Lu Yuanzhen summed up leisure sports as follows: people participate in various sports activities in a voluntary and relaxed mood during their leisure time, and in the process, they can rest their minds and body, relax, and enjoy. Yu Tao regards “leisure sports” as “leisure sports” and defines it as follows: on the basis of the material wealth and spiritual wealth accumulated since the era of industrial society, people actively enjoy and experience sports activities to improve and enrich themselves. A modern form of physical activity brings pleasure. Yu Kehong and Liang Ruowen believe that leisure sports is a modern way of life that individuals carry out through certain physical activities in their free time, to obtain the best psychological experience and a meaningful way. Under normal circumstances, people will choose the content and method of activities independently and pursue the best leisure experience, so that they can relax, satisfy, and enjoy themselves mentally and physically.
3. The purpose of paying attention to leisure sports is to improve the health level: Shi Zhenguo and Tian Yupu define leisure sports as follows: people choose and participate voluntarily in their leisure time, with physical participation as the main way, and the purpose is to restore physical strength and relieve stress, a scientific and healthy way of physical activity for regulating emotions, entertaining the mind and body, and strengthening the body. Xi Yubao, Gao Sheng, and Yang Bin's understanding of leisure sports is that people use their free time at their disposal to independently choose their favorite sports and practice methods to achieve self-cultivation, physical and mental pleasure, self-realization, and self-improvement, a kind of social activity.

RETRACTED

According to the opinions of the abovementioned experts, we define recreational sports as the activities of leisure, health, and leisure and stimulation that individuals participate in during leisure time, knowledge acquisition, and skill improvement and then to gain positive experience.

### 2.3. Development Stage and Characteristics of Leisure Sports Policy Environment in Developed Countries

Western experts have similar views on the evolution of modern leisure sports environment in developed countries such as Britain, the United States, and France. Experts pointed out that the development of the modern leisure sports environment in developed countries has mainly gone through a process: in the initial stage, the government-led policies were vigorously promoted, administrative agencies actively intervened, the government led and social organizations actively led the development and continuous improvement and deepening of modern leisure sports.  Table 2 shows the characteristics of leisure sports in China at different stages.

#### 2.3.1. The Initial Government Guidance Stage Accompanying the Industrial Revolution (Mid-18th Century to Mid-Late 19th Century)

After the beginning of industrial production reform in Western Europe, mass entertainment and sports in the modern sense have taken the lead in the European and American labor class. Therefore, European and American countries have adopted policies and measures to promote and actively promote the vigorous development of leisure sports, so as to avoid social unrest, reduce the criminal rate, and improve social stability. At the initial guidance stage of the policy, the main characteristics of leisure sports in the government environment include the following: (1) leisure sports have not really entered the public supervision line of sight of government departments, and extensive guidance and supervision are the measures taken by government departments to reduce community unrest and criminal crime rate; (2) a number of leisure and fitness venues have been established under the leadership of government departments, but the scale is small, the total amount of activities is small, and the direct investment of government finance is also small.

#### 2.3.2. The Stage of Vigorous Advocacy by the Government before the End of World War II (the End of the 19th Century-the Period of World War II)

During this period, promoting people's leisure sports activities has become a major responsibility of the Chinese government. The state has established leisure public service institutions of the people's government, established leisure and fitness stadiums, and introduced policies and measures to encourage leisure and fitness education activities to promote an active and healthy leisure lifestyle. The important characteristics of the Chinese government's policy environment of vigorously promoting the development of leisure and fitness sports are as follows: (1) the government strongly promotes the development of leisure sports through relevant policies; (2) the main purpose of the Chinese government's actions is not to promote health and economic and social development, but to reduce the crime rate, achieve good social control, and guide the orderly and healthy development of the economy and society.

RETRACTED

#### 2.3.3. The Stage of Systematic Government Intervention after the End of World War II (End of World War II-Late 1970s)

Leisure sports also started in this period, laying a solid foundation for the future high-speed development. This period is often called “leisure welfare period.” Both the central government and the regional governments have carried out all-round intervention in sports and invested huge capital in infrastructure construction. In the policy system intervention stage, the main characteristics of the leisure sports policy environment include the following: (1) the policy intervention scope of local authorities is not only expanding but also becoming more systematic. Various leisure sports laws and regulations have been promulgated and continuously improved, gradually forming an organic system; (2) leisure sports has become an integral part of welfare politics and has been attached to importance by the local government. The state finance has also increased the direct investment in leisure sports.

#### 2.3.4. The Government Guides Social Forces to Dominate the Stage of Leisure Sports (1980s to the End of the 20th Century)

In the 1970s, it was called the era of “sports rights” in Western countries. The Chinese government has made large-scale investment and intervention in sports, but the people are also dissatisfied with the bureaucracy, inefficiency, pollution, and inequality brought by administrative intervention and need to make changes. In developed countries, there was an economic recession in the late 1970s and early 1990s. It is difficult for the government finance to maintain the “huge investment” in sports as in the previous period. Therefore, sports policies such as culture, entertainment, and sports have been restored in a certain sense, and Figure 2 shows the influence of developed country governments on the leisure sports industry.

RETRACTED

#### 2.3.5. The Stage of Continuous Improvement and Deepening in Pursuit of Policy Balance (from the Beginning of the 21st Century to the Present)

In the 21st century, the developed countries have begun to step into the leisure fashion. Entertainment and active entertainment have become the main driving force of national social development. During this period, the preferential policies for entertainment and sports in countries around the world basically inherited the mode of the previous stage and, on this basis, further bridged the differences and gave corresponding preferential policies to key regions and ethnic groups (the elderly, vulnerable groups, patients, disabled persons, women, ethnic minorities, immigrant groups, etc.).

## 3. Development Experience of Leisure Sports Policy Environment in Developed Countries

### 3.1. Government-Led Investment in the Construction of a Large Number of Public Sports Venues and Facilities

The legislation and measures of these countries are clear, and the central government has the task to make a major investment in public sports. The central government expenditure is one of the important sources of public sports expenditure, and the investment of local governments generally exceeds that of the central government. In the 1990s, the financial allocation of British governments at all levels accounted for a certain proportion of the total government input: Germany, England, and Switzerland all accounted for more than 90%, Sweden, Denmark, and Finland all accounted for about 80–90%, and France, Belgium, and Spain accounted for about 70–80%. Although London also has many sources of sports funds, the government still occupies a dominant position in terms of financial resources. In 2009, the total government funding for community and sports undertakings was only 300 million pounds. Among them, the US financial reward fund was 125 million pounds, and the total revenue of the British lottery business was 135 million pounds. The family expenses raised by individuals are as high as 50 million yuan; the financial expenditure on public sports in various regions is even more, exceeding 2 billion pounds per year and increasing at a rate of 4% per year. Local financial investment in leisure sports is mainly concentrated in two areas: ① construction and maintenance of public sports venues and other infrastructure; ② support for sports associations and nonprofit sports clubs.

### 3.2. Use a Higher Proportion of Lottery Funds to Develop Public Sports

In 1994, the sports lottery fund was introduced into public stadiums and was successful. Because this mode is widely dependent on people's “gambling” passion, it can bring stable and lasting investment support. Moreover, in most states, sports lottery funds have also brought a very large proportion of capital investment to public sports. Some developed countries have upgraded these preferential policies to the level of national legislation to protect them. For example, Canada has approved the national development sports lottery law, and Japan has approved the sports lottery law. According to sales statistics, 28% of the total revenue of sports lottery in the developed countries in the UK is used for charity, and about 16.67% is used for sports. From 1994 to 2000, the British government invested about 1.12 billion pounds in sports lottery, exceeding the total amount supported by the Ministry of Finance.  Figure 3 shows the government's investment in leisure sports in developed countries.

RETRACTED

### 3.3. Actively Guide Social Forces and the Market to Develop Leisure Sports Together

Since the 1980s, the national leisure and sports policy has also undergone great changes. The central government has also gradually returned to the “behind the scenes,” mainly to carry out macrocontrol, and social forces have gradually moved to the “front stage,” forming the leading force of local governments. This pattern has been maintained until now. In 1988, the mandatory bidding regulations of the United Kingdom created the “first” market to encourage social funds to flow into entertainment and sports. Since then, all parts of the country have competed to imitate, and the government has become a 0.5 invisible person, whose responsibility is to maintain social fairness and ensure the protection of public sports. Rights and interests: therefore, the state has formulated many regulations and measures to guide the society to invest in the sports industry.

### 3.4. Vigorously Support Grassroots Nonprofit Recreational Sports Clubs

The main service entity of leisure sports institutions in developed countries has a large number of community clubs. This kind of movement organization has a high degree of autonomy and can exclude political functions and obtain tax concessions. The latter includes nonprofit clubs and enterprise clubs. The former usually receives a large amount of financial support and uses public sports venues and other infrastructure at no cost or at low cost, most of which can be donated by the public. In 2012, there were about 91000 sports associations in Germany, with members accounting for more than 1/3 of the total. All nonprofit associations are basically exempt from tax.

### 3.5. Attach Importance to and Actively Guide the Combination of Leisure Sports and Basic Education

The state attaches great importance to providing support for teenagers to establish lifelong sports interests through education. In some countries, school sports, sports events, extracurricular sports, outdoor hiking and camping, school sports hobby organizations, and youth associations are well developed, and sports events and organizations are also very popular in schools. The British government has introduced various measures to improve the relationship between sports clubs or social sports centers and schools. Club members of these schools enjoy discounts. At the same time, the club also cooperates with the college in sports, training, and activities. In 2015, the Australian federal government put forward the action plan of “Sports School.” One of its features is to link the school with sports clubs to complete the transformation between campus sports and social sports. The research results show that more than 70% of American adult outdoor sports enthusiasts have received outdoor sports training in primary schools, which has become one of the main factors for them to continue outdoor sports after they grow up.

RETRACTED

## 4. Implications for the Development of My Country's Leisure Sports Policy Environment

### 4.1. Problems Existing in My Country's Leisure Sports Policy Environment

After the reform and opening up, especially through the efforts of nearly 20 years, China's economic productivity and the quality of people's life have been qualitatively improved. Since the mid-1990s, the leisure demands of Chinese urban residents have increased significantly; due to the implementation of the five-day work week and the eight-hour work day, a large number of sports venues and sports clubs have been created in the city, and leisure sports have flourished. To meet the social needs, various laws, regulations, and measures to promote the rapid development of leisure sports will be promulgated and implemented as soon as possible. Generally speaking, the current legal conditions still lag behind the social reality and have not produced a good driving effect on the rapid development of leisure sports, which is reflected in the following: (1) the policy is more industrialization than welfare; (2) some policies are too general and not specific enough; (3) there are many deficiencies in policies and regulations, and there are no specifications for the definition of specific responsibilities, government supervision, and performance appraisal; (4) supplement, amendment, and abolition of the project are lagging behind; for example, the formulation of current sports laws and regulations is lagging behind; various financial mismatches are common. There are also shortcomings: the intensity, mode, and effect of financial investment need to be optimized; the support of social capital and sports clubs needs to be improved; the high price of leisure sports consumption affects the enthusiasm of public participation; there is an urgent need to promulgate laws and regulations on determining the responsibility of outdoor sports and entertainment safety and thoroughly implement the policies related to recreational sports.  Figure 4 shows various factors affecting the development of leisure sports in China.

RETRACTED

### 4.2. Suggestions for Optimizing the Policy Environment of Leisure Sports in My Country

#### 4.2.1. Adjust the Distribution Method, Intensity, and Direction of Government Direct Investment

With reference to the arrangement method of the national sports fund, we will greatly increase the financial support for leisure sports and adjust the proportion of financial support in the national physical training plan and the Olympic glory plan. It is suggested to reform the distribution mode of national welfare lottery and sports lottery public welfare fund to increase the support for leisure sports. According to the current use of funds of China sports lottery companies, all sports lottery public welfare funds should be used for entertainment sports (at present, the ratio of sports lottery public welfare funds to leisure sports and competitive sports in China is about 6 : 4), and the larger national welfare lottery public welfare funds are all used for entertainment sports. Some of the funds are used for competitive sports.  Table 3 shows the Chinese government's capital investment in leisure sports from 2010 to 2018.

#### 4.2.2. Improve Support for Social Capital and Sports Clubs

The social funds in developed countries are much higher than the national financial investment in entertainment and sports, and they are the “main body” of government organization and management. China should fully mobilize the enthusiasm of the whole society, especially the capital, and extensively participate in the development of recreational sports. To this end, it is necessary to accelerate the transformation of government functions, continue to promote the reform of “relaxing rights, implementing rights, and improving services,” further promote the negative responsibility list management mode, minimize preintervention, and strengthen postevent management; increase local preferential policies to ensure the continuous stability of policies; guide social funds to invest in the construction of infrastructure for recreational sports stadiums, support the development of leisure sports clubs, gradually expand the strength of local preferential policies in land use, taxation, water, and electricity charges, and even directly provide state financial subsidies; and guide social funds to invest in sports events.

RETRACTED

#### 4.2.3. Promulgate Laws and Regulations on the Determination of Liability for Outdoor Sports and Recreational Accidents

The specific requirements for the responsibility of safety accidents in this area shall be formulated, and the specific requirements for the identification of outdoor sports injury responsibility shall be explained in the amendment of sports laws and regulations. The successful experience of developed countries is referred, and the interests of outdoor sports organizers, sponsors, and peers are safeguarded. At the same time, we will improve the compensation system for outdoor sports events. Economic compensation will be realized by social insurance and commercial insurance. Meanwhile, law enforcement and supervision on insurance claims will be strengthened.

#### 4.2.4. Lower the Price of Leisure Sports Consumption and Reduce the Cost of Participation

The scale of free parks in the city is expanded, especially large theme parks. The charges for scenic spots are reduced, or the charging measures for some low-level scenic spots are abolished; tourists who take part in sports exercises in a scenic spot for many times in a year will be given a corresponding discount. The tolls and fuel costs of routes are reduced, the tolls of routes that have exceeded the set tolling period are reduced, and illegal and arbitrary tolls on local roads are prohibited. On the basis of strictly restricting the price of leisure sports venues, the government should reduce the cost of public construction by compensating the price of sports venues or clubs.  Figure 5 shows the per capita consumption of leisure sports in my country.

## 5. Conclusion

The public health system needs to strengthen the relevant legal system and policy environment for protecting health and ensuring safety, so as to lead and regulate the operation and development of the public health system. Through organizational guarantees, the responsibilities and tasks of all parties in the system are clarified; the structure and work process within the organizational system are established; various public health management mechanisms such as planning, monitoring, evaluation, leadership, and coordination are used to improve the health of the population; the human, financial, material, and information resources of public health are combined; the corresponding theoretical methods, technical means, and interventions are continuously improved; and then a support system is established to maintain the effective operation of the system. Foreign leisure sports belongs to the category of large leisure research. It is developed and prospered in the 1960s. After the 1980s, it continued to innovate and integrate and formed urban leisure sports development models with different characteristics. My country's leisure sports research has continued to heat up under the catalysis of a series of top-level designs. After more than 20 years, it can be described as fruitful. The emergence of leisure sports is the symbol and product of the progress of the times. As an important field for the occurrence and development of leisure sports, cities have received attention from all walks of life and have become a new trend in the field of leisure and sports research. In this study, the development stage and characteristics of leisure sports policies in developed countries are described in detail, and by analyzing the development experience of leisure sports policy environment in developed countries, it analyzes the main problems existing in the development of leisure sports policy environment in my country, including policy bias. Industry neglects welfare; some policies are too general, not specific enough, difficult to implement, etc. In response to these problems, with the help of the development experience of developed countries, corresponding strategies are proposed, including national level, social perspective, and legal aspects.

RETRACTED

## Figures and Tables

**Figure 1:** Development of leisure sports in various regions of my country.

**Figure 2:** Influence of developed country governments on the leisure sports industry.

**Figure 3:** Investment in leisure sports in developed countries.

**Figure 4:** Influencing factors of the development of leisure sports in my country.

**Figure 5:** Consumption of leisure sports in my country.

**Table 1:** Characteristics of different leisure sports types.

Type	Segment type	Describe
Gymnasium-type sports service complex	Competition-oriented	Taking the large stadium as the carrier
	National fitness-oriented type	Taking small and medium gyms as carriers
Commercial space carrier-type sports service complex	Sports service-oriented	Taking sports as the main element of the commercial space carrier
	Sports service introduction type	Taking the commercial complex as the carrier
Outdoor sports leisure space sports service complex	Sports tourism	Relying on natural ecological resources
	Fitness and leisure park type	Relying on the space covered by various sports parks
	Sports wellness	Relying on health resource space
Other types of sports service complex	Sports service complexes not covered by the above categories	

RETRACTED

**Table 2:** Characteristics of leisure sports in my country at different stages.

Evolutionary stage	Evolutionary features
Start-up	Starting from scratch, a few independent and scattered homogeneous small enterprises gradually form agglomerations through strengthening connections
Growth period	On the basis of the initial stage, it has developed rapidly, and the system has improved in both quality and quantity
Maturity	The growth rate has slowed down compared with the previous period, and the competition within the leisure sports industry ecosystem has intensified
Stable period (decline period)	In the entire system architecture, the scale is relatively stable

**Table 3:** Chinese government's capital investment in leisure sports from 2010 to 2018.

Years	Government investment in leisure sports industry (100 million yuan)	Financial expenditure (100 million yuan)	Government investment intensity
2010	217.84	89874.16	0.0024
2011	297.04	109247.79	0.0027
2012	352.75	125952.79	0.0028
2013	244.77	140212.1	0.0017
2014	270.42	151785.56	0.0018
2015	303.38	175877.77	0.0017
2016	344.5	187755.21	0.0018
2017	290.1	203085.49	0.0014
2018	290.1	220904.13	0.0013

## Data Availability

The labeled data set used to support the findings of this study is available from the corresponding author upon request.
